# The Effect of Interval Training on the Displacement Speed of Male Good Boxers

**DOI:** 10.1155/2022/1431615

**Published:** 2022-07-30

**Authors:** Yun Hou, Xiangui Bu

**Affiliations:** School of Competitive Sports, Shandong Sport University, Rizhao 276800, China

## Abstract

The change of boxing competition rules has put forward higher requirements on the speed quality of male boxers. To investigate the effect of interval training on the displacement speed of male outstanding boxers and to provide a theoretical basis for targeted improvement of speed quality of male boxers. A 4-week interval training intervention was conducted on 20 male boxing athletes through literature method, interview method, and experimental method. The subjects in the experimental group had higher test results than the control group test data after the experiment, and the test results of the experimental group reached a highly significant difference before and after the experiment, and the test results of the control group before and after the experiment were improved but not significantly different. The effect of interval training was more effective than traditional physical training in improving the displacement speed of male good boxers, which significantly improved the displacement speed of the subjects.

## 1. Introduction

The new rules of boxing make boxing more confrontational, and the special requirements for boxers' speed and power are enhanced. Fast movement, fast punching, and fast change of direction are crucial for boxers to control the pace of the game, fight for the initiative and win the game. The improvement of displacement speed can effectively control the distance with the opponent, so as to fight for the initiative, and the rapid movement after the active attack can make the opponent's counterattack fall short, and the rapid change of direction after the defensive counterattack can create more offensive opportunities. Through literature review, there is a lack of research on boxers' displacement speed by domestic and foreign scholars, and there is a gap in the research on boxers' displacement speed. Relevant studies found that through different types of interval training, boxers' displacement speed can be effectively developed, and through strict control of the rest time between sets, it is beneficial for boxers to better perform good technical movements in a fierce confrontation game environment [1,2], and interval training is a medium-to high-intensity training method, which is similar to the intensity of boxing matches and has an important role in the improvement of athletes' physical functions. Therefore, it is important to study whether interval training has an effect on the displacement speed of good male boxers and to provide a theoretical basis for the training of displacement speed of good male boxers.

## 2. Research Object and Method

### 2.1. Research Subjects

The effect of interval training on the displacement speed of male good boxers was taken as the research object, and 20 male good boxers were selected as the experimental subjects according to the research needs.

### 2.2. Research Methods

#### 2.2.1. Literature Method

We checked the keywords and topics of interval training, displacement speed, and boxers' displacement speed on the Internet, Vipshop, and Wanfang, as well as international academic platforms, to clarify the definition and connotation of interval training and displacement speed, and to organize and summarize all kinds of literature.

#### 2.2.2. Interview Method

According to the needs of the study, in-depth interviews were conducted with 5 experts in athletic training and 5 outstanding boxing coaches, all 10 of whom were working in sports colleges and universities with positive senior titles, to solicit their opinions on the development of interval training programs and the selection of displacement velocity test indexes to provide theoretical guidance for this paper.

#### 2.2.3. Experimental Method

Twenty male outstanding boxing athletes were selected as experimental subjects. The 20 athletes were randomly divided into two groups, 10 in the control group and 10 in the experimental group, the control group used the conventional training method, and the experimental group used the interval training without affecting the conventional training method while integrating interval training into the training for intervention, and the displacement velocity test data of the athletes in the two groups before and after the experiment were compared respectively, and the relevant data were analyzed through the experimental results.

As shown in Table 1, the mean age of the two groups was 20.2 years for the control group and 20.1 years for the experimental group, and the weight data were 69 kg for the control group and 68.4 kg for the experimental group. the height data were 176.1 cm for the control group and 173 cm for the experimental group. *p*-values were 0.79, 0.93, and 0.27, respectively, and the data were not significantly different from each other. *p* > 0.05, and subsequent experimental comparisons could be made.

*Experimental Time and Location*. The experimental period was April 29, 20–2 - May 29, 2022, a total of 4 weeks of experimentation, two training sessions per day, 120 minutes per training session, and 30 minutes of the interval training program was used in each session. The experimental s'te's was the boxing gym of Shandong Sports Institute.

*Experimental Control*. As shown in Table 2 and Table 3, the physical quality training part of the 10 experimental groups was an interval training program, and the physical quality training part of the control group was regular training, and the training content was basically partially the same, and the equipment site was checked and placed well before the experiment, and the experiment was observed well.

*Training center rate control*. The heart rate was controlled at 170–180 beats/min during training, and the heart rate reached 120–140 beats/min after resting between sets before the next set of training.

*Experimental test method and test index*. As shown in Table 4, The displacement speed of boxers refers to the ability of the athletes to change their footwork rapidly or the number of times the athletes move their footwork distance and change within the specified time [1]. The ability of displacement speed is high or low is judged from the shortest time to complete the unit distance, displacement speed is divided into two kinds; linear displacement speed and nonlinear displacement speed. Linear displacement velocity is mainly the velocity of linear and arc displacement, such as 50 m, 100 m, and 200 m. Nonlinear displacement velocity mainly refers to the folding and multidirectional movement velocity such as multidirectional running, and change of direction movement [2]. Displacement speed is measured as 30 m, 50 m, and 60 m, and a specified number of seconds of accelerated running to test the subject's ability to run fast [3]; in summary, displacement speed test indexes should be developed according to the distance of step movement and the number of transformations as well as 50 m as an example of linear displacement and different distances of foldback class, and the test indexes will be sorted and screened, and the reasonableness of the test indexes will be ensured by scoring and screening by experts.

According to Table 5, experts on the test index scoring opinion displacement speed test index selected as 15 s in situ pace jumping, 20 m folding run, 50 m run, and 10 m slide to carry out experimental testing.

## 3. Research Results and Analysis

### 3.1. Concept Definition

#### 3.1.1. The Concept of Interval Training

In the 1950s, German Reindl and Bechler put forward the theory of interval training, believing that training with a heart rate of 170–180 beats per minute, and then training after intervals until the heart rate reaches 100–125 beats per minute, which is conducive to enhancing heart pump function. Boxing is a typical high-intensity interval sport, and high-intensity interval training is commonly used in boxing special training practice, and it is effective in improving the anaerobic lactic acid tolerance of boxers [4,5], interval training can accomplish more and greater training volume than continuous training, and it is less laborious, which helps to improve cardiorespiratory function and material metabolism and other functions [6].

In summary, interval training refers to a training method that imposes strict requirements on the combination of movements, the intensity of the load, and the duration of intervals, so that the body is in a state of not recovering well and repeating the exercises. Displacement speed training is fast, high frequency, high intensity, interval training, and boxers displacement speed training in common with the high intensity, instantaneous. Interval training is used to mobilize athletes' body functions and stimulate their potential. Through interval training, boxers' cardiopulmonary function can be improved, and by adjusting the intensity of the training load, various body functions can be significantly changed.

#### 3.1.2. The Concept of Displacement Velocity

Displacement speed refers to the movement of the body as a whole in space, the ability to move quickly, displacement speed can be divided into two kinds: linear displacement speed and nonlinear displacement speed. Linear displacement speed is mainly the speed of linear and arc displacement; nonlinear displacement speed mainly refers to the folding, multidirectional movement speed; linear displacement speed mainly depends on the action frequency and action amplitude; nonlinear displacement speed determinants in addition to the action frequency, action amplitude also need the ability to change the speed and direction of action. In boxing matches, athletes are on the move to attack and defend, fast and sudden movement with boxing attack often plays a surprise effect. When an opponent attacks, fast footwork movement can effectively dodge the opponent's attack. Fast movement can effectively control the pace of the game. The means of practice for developing displacement speed include folding runs and relay runs of different distances, which require the athletes to complete the training at the fastest possible speed, and the content of the movements developed in the training should be similar to the structure of the boxing game [7–9].

### 3.2. Comparative Analysis of Displacement Velocity Data between the Experimental Group and the Control Group before the Subject's Experiment

The comparison of the 15 s pace jump data between the two groups before the experiment is shown in Table 6, the average of the 15 s pace jump data of the experimental group and the control group are 45.6 times and 45.3 times, respectively, the test results of the experimental group are slightly higher than the control group, and the *p*-value of the 15 s pace jump test of the athletes in the two groups is 0.855 by SPSS software. The athletes were at the same level in the 15 s pace jump and could carry out the subsequent experiment.

Table 6 shows the comparison of the 50 m run data of the two groups before the experiment, the average of the 50 m run data of the experimental group and the control group are 8.05 seconds and 8.01 seconds, respectively, and the performance of the control group is better than the experimental group, and the *p*-value of the 50 m run test data of the athletes in the two groups is 0.840 by SPSS software. The two groups of athletes were at the same level in 50 m running and could carry out the subsequent experiments.

Table 6 shows that the average of the 20 m running data of the two groups before the experiment is 5.29 seconds and 5.49 seconds respectively, the experimental group is better than the control group. The two groups of athletes were at the same level in the 20 m folding run and could carry out the subsequent experiments.

Table 6 compares the 10 m straight-line skating data of the two groups before the experiment, the average of the 10 m straight-line skating data of the experimental group and the control group are 4.12 seconds and 4.36 seconds, respectively, the experimental group is better than the control group, and the *p*-value of the 10 m straight-line skating test of the athletes in the two groups is 0.143 *p* > 0.05, and the athletes in the two groups are at the same level. The two groups of athletes were at the same level in 10 m straight-line skating and could carry out the subsequent experiments.

### 3.3. Comparative Analysis of Displacement Velocity Data between the Experimental Group and the Control Group after the Subject's Experiment

Through Table 7 of the two groups in the postexperimental test 15 s pace jumping data comparison that the experimental group and the control group 15 s pace jumping an average of 51.7 times and 46.2 times, respectively, through the data can be seen that the experimental group performance than the control group is higher, the difference between the two 5.5 times, by statistical analysis that *p* < 0.01 two groups there is a very significant difference that the experimental group after the experiment has made significant progress, improve The effect was more obvious than that of the control group.

Table 7 shows the comparison of the 50 m run data between the two groups after the experiment, the average value of the 50 m run for the experimental group and the control group was 7.35 seconds and 7.71 seconds, respectively. The improvement effect was more obvious than that of the control group.

Table 7 compares the data of the two groups in the postexperimental test of the 20 m fold run, the mean values of the experimental group and the control group in the 20 m fold run are 4.99 seconds and 5.40 seconds, respectively. The effect is more obvious than that of the control group.

Table 7 shows the comparison between the two groups in the postexperimental test 10 m slide step data, the average value of 10 m slide step for the experimental group and the control group is 3.70 seconds and 4.21 seconds, respectively. The improvement effect is more obvious than that of the control group.

### 3.4. Comparative Analysis of Subjects' Displacement Velocity Data before and after the Experiment in the Control Group

The results of the 15 s pace jump, 50 m run, 20 m folding run, and 10 m straight-line glide test were 45.30 times, 8.01 seconds, 5.49 seconds, and 4.36 seconds for the control subjects tested before and after the experiment through Table 8. The control group was trained with traditional physical fitness for 4 weeks, and the test indexes of the control group after the training were 46.2 times, 7.81 seconds, 5.40 seconds, and 4.21 seconds. The paired sample *t*-test was calculated using SPSS software for each group data, and the *p*-values were 0.171, 0.096, 0.066, and 0.084, respectively, and the *p*-values of each data were greater than 0.05, which indicated that each test data are not significantly different. This reflects the fact that the control group athletes had an increase in test scores after 4 weeks of traditional physical training but there was no significant difference.

### 3.5. Comparative Analysis of the Displacement Velocity Data of the Experimental Group before and after the Experiment for the Subjects

The results of the 15 s pace jump, 50 m run, 20 m fold run, and 10 m straight-line glide test were 45.60 times, 8.05 seconds, 5.29 seconds, and 4.12 seconds by passing Table 9 pre- and postexperimental tests on the subjects in the experimental group. The experimental group was trained with interval training for 4 weeks, and the test indexes of the experimental group after training were 51.7 times, 7.35 seconds, 4.99 seconds, and 3.70 seconds The data of each group were calculated using SPSS software for paired samples *t*-test, and it was found that the *p*-value was less than 0.01, which indicated that there were highly significant differences in each test data. This reflects that the athletes in the experimental group had a very significant effect in improving their displacement speed test performance after 4 weeks of interval training in the physical fitness section.

## 4. Conclusion

The test data of the experimental group reached a very significant difference, and the performance before and after the test improved significantly, while the test results of the control group improved but did not show a significant difference, so it can be concluded that the interval training in the experimental group training significantly improved the displacement speed of the experimental group, indicating that the training effect of interval training in daily training is more than the traditional physical training on the displacement speed of the subjects The training effect is better.

Through experimental observation, the movement speed of the feet of the experimental group was significantly higher than that of the control group in the actual combat training, and the recovery speed was significantly stronger than that of the control group during the rest time of the round.

## 5. Limitations of the Study

This paper conducted an experimental study on male outstanding boxers, there is no experimental investigation for athletes of different age groups, different sport levels, and different genders, which is the direction of the subsequent research.

Interval training content in the selection of arrangements to consider the athletes because of the different age groups, gender, and other physical external and internal factors to be treated differently.

## Figures and Tables

**Table 1:** Basic information on the physical condition of the control and experimental groups (*N* = 20).

Body information	Control group	Experimental group	*p*
Age (years)	20.2 ± 0.79	20.1 ± 0.88	0.79
Body weight (kg)	69 ± 16.11	68.4 ± 13.16	0.93
Height (cm)	176.1 ± 3.72	173 ± 6.78	0.27

**Table 2:** Interval training program.

Training methods	Training time (sec)	Break duration (sec)	Number of training groups (groups)
1 Fast pace jumping	30	10	6
2 Front straight back straight front swing small dumbbell air strike	30	10	6
3 Fast high leg lift	30	10	6
4 Left and right each 2m distance fast lateral folding run	30	10	6
5 20 kg weight lifting heel	30	10	6
6 Fast half squat jump	30	10	6

**Table 3:** Comparison of training contents between experimental group and control group.

Part	Control group	Number of training groups (groups)	Training time (min)	Rest time (min)	Experimental group	Number of training groups (groups)	Training time (min)	Rest time in group (s)
Preparation part	(1) Preclass routine	1	5	0	(1) Preclass routine	1	5	0
(20 min)	(2) Warm-up activities	1	15	0	(2) Warm-up activities	1	15	0
Basic part	(1) Traditional training content	1	50		(1) Traditional training content	1	50	

(80 min)	(2) Traditional physical training	1	30		(2) Interval training	1	30	
	Push-ups	2	2	1	(1) fast pace jumping	6	0.5	10
	(2) sit-ups	2	2	1	(2) front straight and back straight forward swinging small dumbbell air strike	6	0.5	10
	(3) vertical push-ups	2	2	1	(3) fast high leg lift	6	0.5	10
	(4) deep squat	2	2	1	(4) left and right each 2m distance fast lateral folding run	6	0.5	10
	(5) trot	2	2	1	(5) 20 kg weighted heel lift	6	0.5	10
	(6) pull-ups	2	2	1	(6) fast half squat jump	6	0.5	10
Closing section	1 Stretching and relaxing	1	20	0	1、Stretching and relaxation	1	20	0
(20 min)	Control group				1、Preclass routine			

**Table 4:** Test item selection.

Test items	Test index	Number of items
Linear displacement speed	50 m run, 100 m run, 10 m skid test, 20 m skid test, 5 s acceleration run	5
Folded displacement speed	15 s pace jump, hexagonal test, 20 m folding run, 10 m folding run, 30 s pace jump	4

**Table 5:** Expert test index scoring table.

Test item	Expert rating (10-point scale)
50 m	10
100 m	8
10 m glide	9
20 m glide	8
5 s acceleration run	8
15 s pace jumping	9
50 m	10
Hexagonal test	6
20 m fold run	9
10 m toss	8
30 s pace jump	7

**Table 6:** Analysis of test data of the experimental and control groups before the experiment (*N* = 20).

Test items	Experimental group (*X* ± SD)	Control group (*X* ± SD)	*t*	*p*
15 s pace jumping (times)	45.60 ± 3.53	45.30 ± 2.36	0.188	0.855
50 m run (sec)	8.05 ± 0.51	8.01 ± 0.42	0.207	0.840
20 m folding run (sec)	5.29 ± 0.18	5.49 ± 0.29	−1.748	0.114
10 m straight-line glide (sec)	4.12 ± 0.38	4.36 ± 0.48	−1.604	0.143

**Table 7:** Analysis of test data of the experimental and control groups after the experiment (*N* = 20).

Test items	Experimental group (*X* ± SD)	Control group (*X* ± SD)	*t*	*p*
15 s pace jumping (times)	51.7 ± 3.16	46.2 ± 2.97	3.579	0.006
50 m run (sec)	7.35 ± 0.40	7.71 ± 0.33	−2.599	0.029
20 m folding run (sec)	4.99 ± 0.21	5.40 ± 0.23	−3.725	0.005
10 m straight-line glide (sec)	3.70 ± 0.41	4.21 ± 0.50	−3.409	0.008

**Table 8:** Analysis of test data of control group before and after the experiment (*N* = 20).

Test items	Pre-experiment (*X* ± SD)	After the experiment (*X* ± SD)	*t*	*p*
15 s pace jumping (times)	45.30 ± 2.36	46.2 ± 2.97	−1.489	0.171
50 m run (sec)	8.01 ± 0.42	7.81 ± 0.25	1.861	0.096
20 m folding run (sec)	5.49 ± 0.29	5.40 ± 0.23	2.089	0.066
10 m straight-line glide (sec)	4.36 ± 0.48	4.21 ± 0.50	1.939	0.084

**Table 9:** Analysis of test data of the experimental group before and after the subject's experiment (*N* = 20).

Test items	Pre-experiment (*X* ± SD)	After the experiment (*X* ± SD)	*t*	*p*
15 s pace jumping (times)	45.60 ± 3.53	51.7 ± 3.16	−7.810	≤0.001
50 m run (sec)	8.05 ± 0.51	7.35 ± 0.40	5.371	≤0.001
20 m folding run (sec)	5.29 ± 0.18	4.99 ± 0.21	7.310	≤0.001
10 m straight-line glide (sec)	4.12 ± 0.38	3.70 ± 0.41	8.466	≤0.001

## Data Availability

The data used to support the study are included in the paper.
